RETRACTED

# A Game Model for Incentive Mechanism of Distributed Nodes in Supply Chains

**DOI:** 10.1155/2021/7502860

**Published:** 2021-12-07

**Authors:** Jingjing Jiang, Aobo Lyu

**Affiliations:** ^1^School of Business, Beijing Union University, Beijing, China; ^2^School of Public Administration, Sichuan University, Chengdu, China

## Abstract

This study aims to solve the credit problems in the supply chain commodity and currency circulation links from the perspective of the ledger, while the game model method has been adopted. The research firstly reviews the relationship between distributed ledger technology and the essential functions of currency. Then, by constructing two-agent single-period and multi-period game models in the entire supply chain, the researchers analysed the incentive mechanism and equilibrium solution of distributed nodes of Central Bank Digital Currency (CBDC). The results of this study include the incentive mechanism and optimization of distributed nodes based on licensed distributed ledger technology, which is an important issue that CBDC faces when performing currency functions. The implications of this study mainly cover the limitations of the underlying technology of the public chain and its reward mechanism in the supply chain management and provide support for the rationality of the CBDC issuance mechanism based on state-owned commercial banks, which provides a reference for the CBDC practice. The main value of the research not only serves the decision-making department of the CBDC issuance but also provides ideas on the operation mode of digital currency for the field of digital currency research.

## 1. Introduction

At present, the global macroenvironment is complex and severe, economic growth has fallen, commodity prices have risen, epidemic trends and economic trends have become complex, and risks and challenges continue. In this context, complying with the digital development trend and doing an excellent job in commodity quality management in a long-term and reliable way has become an essential topic in supply chain management.

Commodity quality management and credit issues have long been concerns in the research field of supply chain management. Although studies have shown that information sharing between supply chains can significantly improve product quality and business performance [1], and producers can contract design and revenue distribution mechanisms to avoid immoral behavior of suppliers [2]; there is still a gap in the research on the authenticity guarantee of credit and commodity quality at the technical level. Some studies have pointed out that blockchain is a new and revolutionary technology that significantly affects the supply chain network and discussed the significance of blockchain technology in supply chain management [3, 4]. Therefore, nowadays, with the innovation and development of distributed ledger technology and its application in Central Bank Digital Currency (CBDC) research and development, using CBDC to support information sharing activity and solving credit and commodity quality management problems in the supply chain scenario has gradually become possible.

RETRACTED

Distributed ledger technology can express rules through algorithm programs to enable participants to trust standard algorithm programs and establish mutual trust in the R & D and application of CBDC to solve the trust problem of commodity quality management in the supply chain scenario with higher efficiency and lower cost. This study intends to take this as the research goal, build a game model to simulate the incentive selection of distributed nodes in distributed ledger technology, and obtain the optimal trusted manager of commodity quality by analyzing the equilibrium solution, to provide a reference for the application of distributed ledger technology in supply chain management and CBDC practice.

The follow-up structure of this paper is organized as follows.  Section 1 discusses the theoretical basis for the possible realization of the function of digital currency by distributed ledger technology and briefly describes its optimization mechanism for the existing currency and how to use distributed ledger technology to realize the function of currency and what problems to be solved urgently.  Section 2 analyses digital currency's incentive and restraint mechanism based on distributed ledger technology by constructing a game model.  Section 3 attempts to solve the equilibrium conditions and puts forward the optimal digital currency distributed nodes selection.  Section 4 is the conclusion of this paper.

## 2. Related Works

### 2.1. Overview of Distributed Ledger Technology

Distributed ledger technology is based on cryptography. Designing and implementing the “consensus” mechanism in multiple distributed nodes can completely and accurately record the complete historical process of transactions and payments. The ledger based on the distributed ledger technology is a publicly visible decentralized shared ledger. “Consensus” is a necessary condition for the distributed ledger to achieve the consistency of multinode records, the robustness of consensus protocols, the efficiency of reaching a steady state through high-speed convergence, and the security of the system [5]. From the technical perspective, the currently recognized consensus mechanisms include proof of work (POW), proof of stake (POS), PBFT, RSCoin, hybrid consensus, and consensus mechanism based on DAG technology.

RETRACTED

### 2.2. Currency Function under Licensed Distributed Ledger Technology

Under the licensed distributed ledger technology, each transaction and payment is updated to the ledger by the licensed distributed node. A consensus is reached through confirmation if it is confirmed as a real transaction or payment by an absolute majority. Among them, how to design the absolute majority protocol to ensure that the distributed node data changing with the transaction and payment is confirmed by the absolute majority protocol and finally reach an agreement, that is, the “consensus” mechanism. At present, it has been used in security settlement systems, trade settlement systems, central bank digital currency design, and “stable currency.”

In a single transaction and payment, the specific process is as follows: different licensed distributed nodes update the ledger according to their respective transactions and payments. Each update needs to be confirmed by an absolute majority of agreements. If it is confirmed as a real transaction and payment, it will be updated in the decentralized shared ledger (DSL). The working principle of the licensed distributed ledger technology is shown in Figure 1.

In society's transactions and payments, smart contracts will record the transactions of goods and services and the receipt and payment process of funds. The use of smart contracts facilitates the recording and verification of distributed ledgers. For manufacturers that generate inferior products and provide inferior services mixed in the transaction and payment process, most nodes of the licensed distributed ledger will verify and update the information and provide the information to the fund payer for decision-making. The working principle of licensed distributed ledger technology in social transactions and payments is shown in Figure 2.

The main role of distributed ledger technology in performing monetary functions is to prevent “double flowers.” All transactions and payments, either using traditional online or offline modes or equipped with smart contracts, can be verified by licensed nodes using distributed ledger technology to avoid the “double flower” problem. The transactions and payments under the distributed ledger technology are recorded through cryptography technology. We can know whether the historical records have been tampered with by encryption and decryption. If the absolute majority is verified to be “true” by the licensed distributed nodes, it proves that the digital currency has not been a “double flower,” and the transactions and payments are effective.

### 2.3. Problems Faced by Digital Currency Performing Monetary Function Based on Distributed Ledger Technology

#### 2.3.1. How to Select Distributed Nodes?

Under the unlicensed distributed ledger technology, any willing and capable economic individual can act as a distributed node to update and verify the ledger. The current public chain chooses to use the unlicensed distributed ledger technology. However, the demanders for digital currency involve almost all economic individuals, and the number of transactions and payments is vast. Each transaction and payment need to be confirmed based on the absolute majority of the consensus mechanism. It takes a lot of computing power under the distributed ledger technology without a license. At the same time, considering the rapid layout and development of quantum technology, the tamper-proof function based on a large amount of computing power investment is at risk of being cracked. Therefore, digital currencies with high-security requirements should adopt licensed distributed ledger technology.

RETRACTED

However, even with licensed distributed ledger technology, digital currency still faces the problem of distributed node effectiveness in performing its currency function. Effective distributed nodes need incentives to provide real authentication information to achieve antitampering and avoid “double flowers.” For licensed distributed nodes, it is difficult to technically ensure that they fully participate in the verification and signature of each transaction, and it is also difficult to technically prohibit them from verifying multiple account books with conflicting accounting items. Because of this, how to select the desired distributed nodes to correctly select and verify the “right” ledger and the “wrong” ledger?

#### 2.3.2. How to Design Incentive Mechanism?

How to design an incentive mechanism to ensure the integrity and authenticity of verification for acceptable licensed distributed nodes? The selected distributed nodes can provide real authentication information and ensure that each transaction can be verified. In addition, how to design a better incentive mechanism so that the verification process of distributed nodes can promote the improvement of transaction scale and quality in the economy?

In this regard, Nosal and Rocheteau [6] proposed that if distributed nodes can publicly obtain historical transaction data, they will have less motivation to make false verification. At the same time, due to reducing the verification cost, it may improve the integrity of verification. Furthermore, the disclosure of historical transactions can help promote the completion of transactions to promote economic growth and high-quality development. However, historical transaction data cannot be obtained completely and in real time [7]. How to design an effective incentive mechanism under the condition of incomplete information so that the income obtained by the information verifier is greater than the cost so that the distributed nodes can provide “pair” verification and verify each transaction and improve the transaction scale and quality at the same time? What is included in the incentive mechanism?

RETRACTED

## 3. Methods

### 3.1. Model Overview

The unlicensed distributed ledger technology may be more vulnerable to historical tampering attacks based on the above analysis. Therefore, the model constructed in this paper should be based on licensed distributed ledger technology. At the same time, under the assumption of incomplete information, an incentive mechanism should be constructed to enable the desired distributed nodes to provide “right” verification as the verifier of transaction information to verify each transaction and improve the decision-making of transaction scale and quality. Therefore, the incentive mechanism should enable the verifier's “verification of” to be partially observed and rewarded, and vice versa. In this regard, Carlsson and Damme [8] proposed the research methods of multiagent information incomplete multistage game and global game, which is the modelling method of this research. It is assumed that decision makers can only observe the profit and loss with continuous noise in the game in the economy with incomplete information, and the equilibrium result is unique, which is a research method with high consistency with the research purpose of this paper.

Morris and Shin [9–11] have used this method to make a series of studies on the self-realization mechanism of the financial crisis and put forward policy suggestions according to the equilibrium results. Brown et al. [12], Hakenes and Schliephake [13], He and Manela [14], Schilling [15], and Yang et al. [4] all used game analysis methods to study the liquidity and system stability in the financial field. Some studies have also used game theory to study the interaction between suppliers and sellers in the supply chain [16, 17]. Therefore, this paper intends to build a game model on this basis and design the digital currency transaction verification incentive mechanism and consensus mechanism based on the licensed distributed ledger technology according to the equilibrium results of the model.

### 3.2. Model Assumptions

Based on the working principle of licensed distributed ledger technology in social transactions and payments shown in Figure 2, this study establishes a model to analyze the selection of producers and verifiers. The operation of the model follows the following assumptions.

RETRACTED

**Assumption 1 s 1.**

The whole social production is divided into two stages, and consumers can only obtain utility from the final products or services provided by downstream manufacturers. The producers are divided into stage-I producers and stage-II producers. The former produces raw materials, including upstream and midstream manufacturers in Figure 2, and the stage-II producers produce final products, i.e., downstream manufacturers in Figure 2.

**Assumption 2 s 2.**

In the whole society, consumers are producers. Then, consumers include stage-I producers and stage-II producers, that is, the demander of the final product in Figure 2.

**Assumption 3 s 3.**

Inferior producers and inferior service providers only exist in stage-II producers. This is because the stage-II producers produce the final products, and the stage-II producers consume the final products. Therefore, for the stage-II producers, this group consumes the goods produced or services they provide. Therefore, it is assumed that there is no possibility of producing inferior products or providing inferior services.

**Assumption 4 s 4.**

Based on the licensed distributed ledger technology, since only stage-I producer may choose to produce inferior goods or provide inferior services, only stage-I producer may be involved in whether the confirmed transaction and payment information are “true.” Therefore, it is assumed that the confirmation of whether the transaction and payment information is “true” can only be completed by stage-II producers.

**Assumption 5 s 5.**

The transaction and payment system contain several cycles. In the first production cycle, if the stage-II producer provides false information as the information confirmer, it will be punished by being excluded from the transaction and payment system. Therefore, it is assumed that the stage-II producer will not provide false information in the first production cycle.

**Assumption 6 s 6.**

Each entity makes the current strategy choice according to the historical decisions of other entities.

### 3.3. Model Development

#### 3.3.1. Utility Analysis of Various Subjects

If the proportion of manufacturers' producing inferior products and providing inferior services in the stage I is *f* (*f* stands for fault), the total number of manufacturers in the stage II becomes  1 − *f* (this is because the manufacturers producing inferior products and providing inferior services in the stage I are observed, so they are excluded from the stage-II trading system) of the total number in stage I.

*(1) Stage-I Qualified Producers*. The utility of a qualified producer in stage I comes from the difference between the goods or services enjoyed and the goods or services provided. Therefore, the utility function of a qualified producer in stage I is

(1) $$\begin{array}{c} U_{1}=U_{1}\left[\left(1-f\right)y_{2}\right]-P\left(1-f\right)y_{2}-y_{1}+Py_{1}, \end{array}$$

where *U*_1_ represents the utility function of qualified producers in stage I, *y*_1_ refers to the qualified goods or services produced and sold by producers in stage I, that is, the qualified goods or services consumed by producers in stage II, *y*_2_ means the qualified goods or services produced and sold by the stage-II producer, that is, the qualified goods or services consumed by the stage-I producer, then (1 − *f*)*y*_2_ refers to the qualified goods or services consumed by qualified producers in stage I, *U*_1_[(1 − *f*)*y*_2_] refers to the utility obtained by a qualified producer in stage I from the qualified goods or services consumed by him, *P* represents the general price level of goods or services, *Py*_1_ represents the production income of qualified producers in stage I, and *P*(1 − *f*)*y*_2_  represents the consumption expenditure of qualified producers in stage I.

*(2) Inferior Producers and Inferior Service Providers in Stage I*. The utility of inferior producers and service providers in stage I comes from the qualified goods or services in stage II. Therefore, the utility function of inferior producers and service providers in stage I is

(2) $$\begin{array}{c} U_{1f}=U_{1}\left(fy_{2}\right)-Pfy_{2}, \end{array}$$

where *fy*_2_ refers to the qualified goods or services consumed by inferior producers in stage I, *U*_1_(*fy*_2_) refers to the utility obtained by inferior producers in stage I from the qualified goods or services consumed by them, and *Pfy*_2_ represents the consumption expenditure of inferior producers in stage I.

*(3) Stage-II Qualified Producers*. The utility of the stage-II producer comes from the difference between the utility enjoyed by the qualified goods or services purchased from stage I producer as raw materials and the goods or services provided. Therefore, the utility function of the stage-I producer is

(3) $$\begin{array}{c} U_{2}=U_{2}\left(y_{1}\right)-Py_{1}-y_{2}+Py_{2}, \end{array}$$

where *U*_2_(*y*_1_) refers to the utility enjoyed by the stage-II producer in purchasing qualified goods or services as raw materials from the stage-I producer and *Py*_2_ represents the production income of stage-II producers.

RETRACTED

#### 3.3.2. Game Strategy Selection of Various Subjects

*(1) Stage-I Producers*. At stage I, producers can choose two strategies: one is to produce qualified products or provide qualified services, and the other is to produce inferior products or provide inferior services.

*(2) Stage-II Producers*. According to the analysis of the hypothesis part of this paper, the stage-II producers can only produce qualified products or provide qualified services, so there is no strategy selection in production. As shown in Figure 2, the strategy selection of stage-II producers may occur in the information confirmation stage based on licensed distributed ledger technology. At the same time, according to the analysis of the hypothesis part of this paper, only stage-I producers may choose to produce inferior products or provide inferior services. Therefore, only stage-I producers may involve the confirmed information, which means the stage-II producers can choose two strategies: one is confirmed as “true,” and the other is not confirmed as “true.”

#### 3.3.3. Game Profit and Loss Matrix of Various Subjects

*(1) Profit and Loss Matrix in the First Complete Production Cycle*. In the first production cycle, various entities do not master the historical strategy choices of other entities; especially, the stage-II producers, who undertake the task of information confirmation, are likely to make wrong decisions in the first production cycle. According to the utility analysis of various entities, the following four quadrant profit and loss matrix is obtained, as shown in Table 1.

Profit and Loss Analysis of Each Entity in the First Quadrant. If all stage-I producers choose to produce qualified products or provide qualified services, and stage-II producers, as information confirmers, make correct judgment and confirm it as “true,” the profit and loss obtained by stage-II producers is as follows. *U*_2_(*y*_1_) − *Py*_1_ − *y*_2_+*Py*_2_+*R* refers to the utility enjoyed by qualified goods or services purchased as raw materials from stage-I producers, minus the consumption expenditure paid for this, then excluding the payment for stage-II production, plus the income obtained therefrom and finally plus the remuneration obtained as an information confirmer. The profit and loss obtained by the producer in the corresponding stage I is *U*_1_(*y*_2_) − *Py*_2_ − *y*_1_+*Py*_1_, that is, the utility enjoyed by qualified goods or services purchased from stage-II producers, minus the consumer expenditure paid for this, and then excluding the payment for stage-I production, plus the income obtained therefrom.

Profit and Loss Analysis of Each Entity in the Second Quadrant. If stage-I producer chooses to produce inferior products or provide inferior services, and the stage-II producer, as the information confirmer, makes a wrong judgment and confirms it as “true,” the profit and loss obtained by the stage-II producer is *U*_2_[(1 − *f*)*y*_1_] − *Py*_1_ − *y*_2_+*Py*_2_+*R*, which refers to the utility enjoyed by qualified goods or services purchased as raw materials from stage-I producers minus the consumption expenditure paid for it. Since stage-II producers can only obtain utility from qualified products or services provided by stage-I producers, but do not confirm inferior products, they can only enjoy the utility of 1 − *f* ratio, However, it is necessary to pay for all products or services (including inferior products and services), exclude the payment for the stage-II production, add the income thus obtained, and finally add the remuneration obtained as the information confirmer. The profit and loss obtained by the producer in the corresponding stage I is *U*_1_(*fy*_2_) − *Pfy*_2_+*Py*_1_, that is, the utility enjoyed by qualified goods or services purchased from stage-II producers, minus the consumer expenditure paid for this, plus the income from the provision of all products or services (including inferior goods and inferior services).

RETRACTED

Profit and Loss Analysis of Three Quadrant Entities. If all stage-I producers choose to produce qualified products or provide qualified services, but stage-II producers, as information confirmers, identify the part with proportion *F* as inferior product producers or inferior service providers, and therefore do not confirms it as “true,” the profit and loss obtained by stage II producers is *U*_2_[(1 − *f*)*y*_1_] − *P*(1 − *f*)*y*_1_ − *y*_2_+*Py*_2_+(1 − *f*)*R*, which refers to the utility enjoyed by qualified goods or services purchased from stage-I producers as raw materials, minus the consumption expenditure paid for this, and then excluding the payment for stage-II production, plus the income obtained therefrom. It should be explained that based on the licensed distributed ledger technology if the information is determined not to be “true,” it does not need to be confirmed, so it is impossible to obtain the remuneration of the information confirmer. Therefore, in this case, the stage-II producer only obtains the corresponding confirmation remuneration for the part confirmed as “true.” The profit and loss obtained by the producer in the corresponding stage I is *U*_1_(*y*_2_) − *Py*_2_ − *y*_1_+*P*(1 − *f*)*y*_1_, that is, the utility enjoyed by qualified goods or services purchased from stage-II producers, minus the consumer expenditure paid for this, excluding the payment for stage-I production, plus the income from products or services confirmed as “real.”

Profit and Loss Analysis of Four Quadrant Entities. If stage-I producer chooses to produce inferior products or provide inferior services and the stage-II producer, as the information confirmer, makes a correct judgment and does not confirm it as “true,” the profit and loss obtained by the stage II producer is *U*_2_[(1 − *f*)*y*_1_] − *P*(1 − *f*)*y*_1_ − *y*_2_+*Py*_2_+(1 − *f*)*R*, i.e., the utility enjoyed by the qualified goods or services purchased as raw materials from the producers in stage I, minus the consumption expenditure paid for this purpose and plus the recognition remuneration obtained for the part confirmed as “true.” The profit and loss obtained by the producer in the corresponding stage I is *U*_1_(*fy*_2_) − *Pfy*_2_, that is, the utility enjoyed by qualified goods or services purchased from stage-II producers minus the consumer expenditure paid for this.

*(2) Profit and Loss Matrix in Subsequent Production Cycles*. Under the assumption of adaptive expectation, the stage-II producer as the information confirmer can obtain feedback according to the consumption feeling after the first production cycle and identify and eliminate the inferior producers and inferior service providers from the trading and payment system, so as to adjust the information confirmation in the subsequent production cycle. Based on this, the stage-II producer as the information confirmer may make a wrong judgment because stage-I producer no longer provides qualified products or services and chooses to produce inferior products or provide inferior services. Based on this, the following four-image limit profit and loss matrix for the subsequent production cycle is obtained, as shown in Table 2.

RETRACTED

Profit and Loss Analysis of Each Entity in the First Quadrant. If all the stage-I producers choose to produce qualified products or provide qualified services and the stage-II producers, as the information confirmer, make a correct judgment and confirm it as “true,” the profits and losses obtained by the stage-II producers are the same as those in the first complete production cycle and will not change.

Profit and Loss Analysis of Each Entity in the Second Quadrant. In the first production cycle, the stage-II producers did not exclude the stage-I producers who chose to provide inferior products or services from the trading and payment system, but they were identified after consumption experience. The “missed fish” can only be lucky once. Therefore, in the subsequent production cycle, it is only possible for the stage-I producers to choose to provide inferior products or services, At the same time, the stage-II producer, as the information confirmer, makes a wrong judgment and confirms it as “true.” Therefore, the profits and losses of producers in stage I and stage II of each production cycle remain unchanged, but the individual producers in stage I who choose to provide inferior products or services have changed.

RETRACTED

Profit and Loss Analysis of Three Quadrant Entities. The profit and loss of the three quadrants in the subsequent production cycle are similar to that of the two quadrants. The misjudgment made by the stage-II producer in the first production cycle will be identified afterwards through the consumption experience, and the misjudgment will only occur once. Therefore, in the subsequent production cycle, it can only be a new misjudgment, and the stage-I producer providing qualified products or services is not confirmed as “true.” Therefore, the profits and losses obtained by producers in stage I and stage II of each production cycle remain unchanged, but the misjudged individuals have changed.

Profit and Loss Analysis of Four Quadrant Entities. As the stage-II producers in each production cycle correctly identify the stage-I producers providing inferior products or services and remove them from the trading and payment system, there should be fewer and fewer stage-I producers actively choosing to provide inferior products or services; then, the profit and loss obtained by the stage-II producers is *U*_2_[(1 − *f*)^*n*^*y*_1_] − *P*(1 − *f*)^*n*^*y*_1_ − *y*_2_+*Py*_2_+(1 − *f*)*R*; the profit and loss obtained by the producer in the corresponding stage I is *U*_1_(*f*^*n*^*y*_2_) − *Pf*^*n*^*y*_2_.

## 4. Results and Discussion

### 4.1. Equilibrium Solution in the First Complete Production Cycle

#### 4.1.1. When Stage-I Producer Provides Qualified Products or Services

For the stage-II producer as the information confirmer, when the stage-I producer chooses to provide qualified products or services, the stage-II producer will choose to make a correct judgment and confirm the production, payment. and transaction information of the stage-I producer as “true.” This is because, from the profit and loss matrix, when *U*_2_(*fy*_1_) − *Pfy*_1_+*fR* > 0, the benefit obtained by the stage-II producer when it is confirmed as “true” is greater, and the utility obtained by the stage-II producer from the stage-I producer must be greater than the expenditure, so *U*_2_(*fy*_1_) > *Pfy*_1_. At the same time, the stage-II producer misjudgment rate *f* > 0, and the information confirmation reward *R* > 0.

Therefore, when the stage-I producer chooses to provide qualified products or services, the stage-II producer will choose to make a correct judgment and confirm the production, payment, and transaction information of the stage-I producer as “true.”

#### 4.1.2. When Some Stage-I Producers Provide Inferior Products or Services

When some stage-I producers provide inferior products or services, whether the stage-II producers can choose to make a correct judgment and not confirm the production, payment, and transaction information of the stage-I producers as “true” depends on the information available to confirm the reward *R*. This is because it can be obtained from the profit and loss matrix when *Pfy*_1_ − *fR* > 0; the income obtained by the stage-II producer when it is not confirmed as “true” is greater, that is, when *R* is smaller, the stage-II producer is more likely to make a correct judgment. However, *R* is the incentive means for stage-II producers as information confirmers. If *R* is too small, stage-II producers lack the incentive to confirm information.

RETRACTED

Therefore, when some stage-I producers provide inferior products or services, stage-II producers may not be willing to become information confirmers, or it is difficult to make a correct judgment, and the production, payment, and transaction information of stage-I producers providing inferior products or services are not confirmed as “true.”

#### 4.1.3. When the Stage-II Producer Confirms the Information as “True”

When the stage-II producer confirms the information as “true,” the stage-I producer will choose to provide inferior products or services. This is because, from the profit and loss matrix, when*U*_1_(*y*_2_) − *Py*_2_ − [*U*_1_(*fy*_2_) − *Pfy*_2_] − *y*_1_ < 0, the income of producers providing inferior products or services in stage I is greater. According to the principle of diminishing marginal utility, the difference between the utility and expenditure of producers in stage I decrease with the increase of consumption, and the above inequality is true.

#### 4.1.4. When the Stage-II Producer Does Not Confirm the Information as “True”

When the stage-II producer does not confirm the information as “true,” whether the stage I producer chooses to provide inferior products or services depends on the rate  *f* that the stage-II producer thinks it provides inferior products. This is because, from the profit and loss matrix, when *U*_1_(*y*_2_) − *Py*_2_ − [*U*_1_(*fy*_2_) − *Pfy*_2_] − *y*_1_+*P*(1 − *f*)*y*_1_ < 0, the income of producers providing inferior products or services in stage I is greater. According to the principle of diminishing marginal utility, the difference between the utility and expenditure of producers in stage I decreases with the increase of consumption. At the same time, the greater *F*, the greater the possibility of the above inequality.

That is, failure to confirm the information as “true” will bring incentives for producers in stage I to provide inferior products or services.

RETRACTED

#### 4.1.5. Analysis of Equilibrium Solution in the First Complete Production Cycle

According to the above analysis, based on Hypothesis 4, the stage-II producers should be given a certain information confirmation reward as an incentive. At this time, confirmed as “true,” providing inferior products or services is the Nash equilibrium of the game matrix, and the profit and loss combination at this time is *U*_2_[(1 − *f*)*y*_1_] − *Py*_1_ − *y*_2_+*Py*_2_+*R* and *U*_1_(*fy*_2_) − *Pfy*_2_+*Py*_1_.

Under the Nash equilibrium, the stage-II producers who only consider the current income have more incentive to confirm the information as “true” and obtain corresponding remuneration. The stage-I producers who only consider the current income will partially tend to provide inferior products or services, so as to enjoy the income from selling products or providing services, but pay less costs. It can be seen that the incentive mechanism should be optimized for the short-sighted behavior of various subjects, and the long-term equilibrium should be solved by constructing a multiproduction cycle game model.

### 4.2. Equilibrium Solution in Subsequent Production Cycles

#### 4.2.1. When Stage-I Producer Provides Qualified Products or Services

When the producers in stage I choose to provide qualified products or services, the profit and loss matrix is in the same form as the first production cycle, so the equilibrium point is also the same. The producers in stage II will choose to make a correct judgment and confirm the production, payment, and transaction information of the producers in stage I as “true.”

That is, when the stage-I producer chooses to provide qualified products or services, the stage-II producer will choose to make a correct judgment and confirm the production, payment, and transaction information of the stage-I producer as “true.”

#### 4.2.2. When Some Stage-I Producers Provide Inferior Products or Services

When some stage-I producers provide inferior products or services, whether the stage-II producers can choose to make a correct judgment and not confirm the production, payment, and transaction information of the stage-I producers as “true” depends on the ratio *F* of the stage-I producers providing inferior products or services and the information confirmation reward *r* available. This is because, from the profit and loss matrix, when *U*_2_[(1 − *f*)^*n*^*y*_1_] − *U*_2_[(1 − *f*)*y*_1_] − *P*(1 − *f*)^*n*^*y*_1_+*Py*_1_ − *fR* > 0, the income obtained by the stage-II producer is greater when it is not confirmed as “true,” that is, when *f* and *R* are small, the stage-II producer is more likely to make a correct judgment. However, similarly, the size of *f* is difficult to control, and too small *R* will lead to the lack of incentive of confirmation information for stage-II producers.

RETRACTED

Therefore, when some stage-I producers provide inferior products or services, stage-II producers may not be willing to become information confirmers, or it is difficult to make a correct judgment, and the production, payment, and transaction information of stage-I producers providing inferior products or services are not confirmed as “true.”

#### 4.2.3. When the Stage-II Producer Confirms the Information as “True”

When the stage-II producer confirms the information as “true,” the profit and loss matrix is the same in form as the first production cycle, so the equilibrium point is also the same. The stage-I producer must choose to provide inferior products or services.

#### 4.2.4. When the Stage-II Producer Does Not Confirm the Information as “True”

When the stage-II producer does not confirm the information as “true,” whether the stage-I producer chooses to provide inferior products or services depends on how many production cycles in the stage-II producer acts as the information confirmer and the ratio  *f* that the stage-II producer believes it provides inferior products. This is because, as can be seen from the profit and loss matrix, if the stage-II producer acts as the information confirmer for a long time, there may be insufficient consumption in the economy due to the elimination of too many stage-I producers in the transaction and payment system; *U*_1_(*y*_2_) − *Py*_2_ − [*U*_1_(*f*^*n*^*y*_2_) − *Pf*^*n*^*y*_2_] may be negative first and then positive, but with the increase of the rate *f* that stage-II producers think stage-I producers provide inferior products, the value of −*y*_1_+*P*(1 − *f*)*y*_1_ will also decrease; then, *U*_1_(*y*_2_) − *Py*_2_ − [*U*_1_(*f*^*n*^*y*_2_) − *Pf*^*n*^*y*_2_] − *y*_1_+*P*(1 − *f*)*y*_1_ < 0 is more likely to be established.

That is, failure to confirm the information as “true” and acting as the information confirmer for a long time will bring incentives for producers in stage I to provide inferior products or services.

#### 4.2.5. Analysis of Equilibrium Solution in Subsequent Production Cycle

According to the above analysis, confirmed as “true,” providing inferior products or services is the Nash equilibrium of the game matrix, and the profit and loss combination at this time is *U*_2_[(1 − *f*)*y*_1_] − *Py*_1_ − *y*_2_+*Py*_2_+*R* and *U*_1_(*fy*_2_) − *Pfy*_2_+*Py*_1_.

Under the Nash equilibrium, the stage-II producers have more incentive to confirm the information as “true.” As they act as information confirmers in multiple production cycles, the stage-II producers have more incentive to confirm the transactions and payments of “right.” Of course, at the same time, the producers of false transactions and payments are excluded, and they will be rewarded if they are confirmed as “true.” In stage I, producers will partially tend to provide inferior products or services, so as to enjoy the income from selling products or providing services, but pay less costs.

RETRACTED

### 4.3. Better Selection of Distributed Nodes

From the above multiperiod game analysis and equilibrium results of incomplete information, it can be seen that, from the perspective of individual participants, if the stage-II producer acts as the information confirmer, it will face the contradiction of whether it acts as the information confirmer for multiple consecutive periods: if it acts as the information confirmer only in a few production cycles, it is possible to confirm too much as “true” to obtain remuneration. If you act as an information confirmer in consecutive production cycles, there is a risk of insufficient consumption in the economy. At the same time, producers at stage I are also vulnerable to incentives to provide inferior products or services.

Therefore, a better choice is to try to use trusted financial intermediaries as licensed distributed nodes. Trusted financial institutions represented by systemically important banks have a clear motivation to identify producers who provide inferior products or services and can also avoid the problem of false confirmation as “true” in order to obtain information confirmation remuneration. Under this mechanism, the stage-II producer will no longer act as the information confirmer, but trusted financial institutions such as commercial banks that have more information about the manufacturer will assume the function of confirming the information. The transaction information can be confirmed in the form of associated smart contracts, and the transaction information can be confirmed as “true” if it is consistent with the bank account. The optimization scheme of digital currency distributed nodes based on permitted DLT is shown in Figure 3.

## 5. Conclusion

The relationship between currency and credit is inseparable. Currency must have a good credit foundation. At the same time, currency performs its essential functions relying on credit. With the innovative development of distributed ledger technology, the requirements of currency on credit may be further met. This paper explores the close relationship between currency, credit, and account book and provides a theoretical explanation for solving the credit problem in currency from the perspective of account book. Based on the highly consistent relationship between distributed ledger technology and the essential functions of currency, this paper analyses the incentive mechanism of distributed nodes of digital currency. It obtains the equilibrium solution by constructing two main body single-stage and multistage game models. This study found that if the producer of the final product or the provider of the final service is the most licensed distributed node, it may lead to the risk of over recognition and insufficient consumption in the economy. On this basis, aiming at the above possible problems and combined with the reality of China's digital currency issuance, this paper puts forward the optimal selection of digital currency distributed nodes. It uses trusted financial intermediaries as licensed distributed nodes, providing a reference basis for the research and development of China's digital currency and its practice in economy and finance.

RETRACTED

Therefore, this paper has some contributions to the research in the field of CBDC. Bis [11] and Xiao (2020) have proposed that since CBDC involves huge transaction and payment data, the distributed ledger technology without a license is not applicable when selecting distributed nodes. For this, Nosal and Rocheteau [6] have demonstrated that licensed distributed ledger technology can improve verification integrity. However, for licensed distributed nodes, it is difficult to technically prohibit them from verifying multiple ledgers with conflicting accounting items. This paper agrees with this view and, on this basis, further discusses how to select the distributed node of CBCD to ensure that it can perform the monetary function well and take into account the cost problem, that is, how to select the desired distributed node so that it can correctly select the account book that verifies “right” and the account book that does not verify “wrong.”

In addition, there are still some limitations of this study. This paper puts forward the viewpoint of taking the systemically important commercial bank as the optimally distributed node. This viewpoint is based on the conclusion that the final product producer or the final service provider cannot be the optimally distributed node. Therefore, it still lacks rigorous mathematical inference, which will also be the research direction and focus in the next step. Moreover, because digital currency has not been widely used in any country or region, the conclusion of this paper also lacks the support of empirical data, which will be supplemented in the subsequent stage of research with the continuous application of digital currency.

## Figures and Tables

**Figure 1:** How the licensed distributed ledger technology works?

RETRACTED

**Figure 2:** How the licensed distributed ledger technology works in social transactions and payments?

**Figure 3:** Digital currency distributed node optimization scheme based on permitted DLT.

**Table 1:** Profit and loss matrix of each entity in the first complete production cycle.

		Stage-I producers	
		Produce qualified products	Produce inferior products
Stage-II producers	Confirm it as “true”	*U*_2_(*y*_1_) − *Py*_1_ − *y*_2_+*Py*_2_+*R* and *U*_1_(*y*_2_) − *Py*_2_ − *y*_1_+*Py*_1_	*U*_2_[(1 − *f*)*y*_1_] − *Py*_1_ − *y*_2_+*Py*_2_+*R* and *U*_1_(*fy*_2_) − *Pfy*_2_+*Py*_1_
	Not confirm it as “true”	*U*_2_[(1 − *f*)*y*_1_] − *P*(1 − *f*)*y*_1_ − *y*_2_+*Py*_2_+(1 − *f*)*R* and *U*_1_(*y*_2_) − *Py*_2_ − *y*_1_+*P*(1 − *f*)*y*_1_	*U*_2_[(1 − *f*)*y*_1_] − *P*(1 − *f*)*y*_1_ − *y*_2_+*Py*_2_+(1 − *f*)*R* and *U*_1_(*fy*_2_) − *Pfy*_2_

**Table 2:** Profit and loss matrix of each entity in subsequent production cycles.

		Stage-I producers	
		Produce qualified products	Produce inferior products
Stage-II producers	Confirm it as “true”	*U*_2_(*y*_1_) − *Py*_1_ − *y*_2_+*Py*_2_+*R* and *U*_1_(*y*_2_) − *Py*_2_ − *y*_1_+*Py*_1_	*U*_2_[(1 − *f*)*y*_1_] − *Py*_1_ − *y*_2_+*Py*_2_+*R* and *U*_1_(*fy*_2_) − *Pfy*_2_+*Py*_1_
	Not confirm it as “true”	*U*_2_[(1 − *f*)*y*_1_] − *P*(1 − *f*)*y*_1_ − *y*_2_+*Py*_2_+(1 − *f*)*R* and *U*_1_(*y*_2_) − *Py*_2_ − *y*_1_+*P*(1 − *f*)*y*_1_	*U*_2_[(1 − *f*)^*n*^*y*_1_] − *P*(1 − *f*)^*n*^*y*_1_ − *y*_2_+*Py*_2_+(1 − *f*)*R* and *U*_1_(*f*^*n*^*y*_2_) − *Pf*^*n*^*y*_2_

## Data Availability

The data used to support the findings of the study are available from the corresponding author upon request.
